The article "The Role of Change Rates of CYFRA21-1 and CEA in Predicting Chemotherapy Efficacy for Non-Small-Cell Lung Cancer" was retracted in 2023. Reasons: signs of a paper mill; suspected computer-generated content; unreliable results or conclusions; lack of ethics approval or compliance.

# The Role of Change Rates of CYFRA21-1 and CEA in Predicting Chemotherapy Efficacy for Non-Small-Cell Lung Cancer

**DOI:** 10.1155/2021/1951364

**Published:** 2021-09-21

**Authors:** Tongwei Zhao, Guangyun Mao, Ming Chen

**Affiliations:** ^1^The Second Affiliated Hospital of Soochow University, Suzhou, Jiangsu Province, China; ^2^Oncology Center, Oncology Department, Zhejiang Provincial People's Hospital, Hangzhou, Zhejiang Province, China; ^3^People's Hospital of Hangzhou Medical College, Hangzhou, Zhejiang Province, China; ^4^School of Public Health & Management, Wenzhou Medical University, Wenzhou, Zhejiang, China

## Abstract

**Background:**

Cytokeratin 19 fragment 21-1 (CYFRA21-1) and carcinoembryonic antigen (CEA) are effective prognostic biomarkers for lung cancer. This study investigated the predictive effects of change rates of CYFRA21-1 and CEA before and after the first cycles of chemotherapy on advanced IIIb/IIIc or IV stage non-small-cell lung cancer (NSCLC) patients.

**Methods:**

Data of 103 NSCLC patients who received chemotherapy in Zhejiang Provincial People's Hospital from February 2018 to November 2020 were retrospectively analyzed. All patients received platinum doublet chemotherapy for at least 2 cycles. CYFRA21-1 and CEA levels of patients were detected before and after the first chemotherapy cycle, respectively. After the second cycle, the efficacy was evaluated, and patients were divided into the disease control (DC) and progressive disease (PD) groups. The generalized linear model (GLM) and linear trend test assessed the relationship between change rates of CYFRA21-1 and CEA levels and chemotherapeutic efficacy before and after chemotherapy. Moreover, the receiver operating characteristic (ROC) curve determined the predictive value of change rates of CYFRA21-1 and CEA on chemotherapeutic efficacy.

**Results:**

After the second chemotherapeutic cycle, there were 92 patients in the DC group and 11 in the PD group. GLM and linear trend test both indicated that change rates of CYFRA21-1 and CEA were inversely correlated with chemotherapeutic efficacy for NSCLC. Change rates of CYFRA21-1 and CEA were used to predict area under the ROC curve of chemotherapeutic efficacy (0.87, 0.71-1.00), which is better than single index prediction of CYFRA21-1 (0.71, 0.49-0.94) or CEA change rate (0.85, 0.69-1.00) (*p* < 0.001).

**Conclusion:**

Before and after chemotherapy of the first cycle for advanced NSCLC patients, combining serum CYFRA21-1 and CEA levels could increase sensitivity and specificity to predict the chemotherapeutic efficacy and guide the following therapy of advanced NSCLC patients.

## 1. Introduction

Lung cancer (LC) is a major cause of global deaths [1]. Non-small-cell lung cancer (NSCLC) accounts for 85% of all diagnosed LC cases, and 70% of patients are already in the advanced stage (stage IIIB/IV) at diagnosis [2]. In the last decade, the development of targeted treatment and immunotherapy based on molecular and immunology research offers abundantly available therapy regimens [3]. Chemotherapy develops slowly relative to the above therapies, while evidence has demonstrated its crucial role in NSCLC treatment regardless of the clinical stages, histology, mutation subtypes, and immune status [4]. Furthermore, chemotherapy is also an effective follow-up approach in case of failure of targeted therapy and immunotherapy [5]. Chemotherapy, therefore, remains the most reliable therapy of precision medicine [6]. The National Comprehensive Cancer Network (NCCN) and other clinical guidelines all recommend platinum-based chemotherapy as the first-line and follow-up treatment for NSCLC [7]. Platinum chemotherapy plus immunotherapy is the most widely used first-line treatment for advanced NSCLC without epidermal growth factor receptor (EGFR) mutation or anaplastic lymphoma kinase (ALK) and ROS-1 rearrangement [8]. Nonetheless, the efficacy of chemotherapy is limited, and its cytotoxicity holds adverse effects on the life quality of patients.

Exploration and clinical application of biomarkers are vital strategies not only for early screening of diseases but also for the identification of patients showing significant efficacy during treatment. Abundant studies elaborated that serum tumor markers (STMs) play a crucial role in cancer diagnosis, prognosis prediction, and recurrence monitoring [9, 10]. The invasiveness of tumor biomarkers is less than that of radiation or endoscopy. RECIST 1.1 is the gold standard for imaging-based assessment of the response of patients with cancers to multiple antitumor therapies, such as chemotherapy [11]. However, this system is deficient. On the one hand, patients had to receive at least 2 cycles of chemotherapy before efficacy evaluation, leading to lagged results, which delays treatment plan adjustment. Other problems may also arise, including adverse effect, economic burden, and hospital stay. On the other hand, the assessment scope of RECIST 1.1 is limited for tumors of empty organs, serosal effusion, and bone metastasis. On the contrary, serum tumor markers are independent of detection time and tumor location. It can be used to predict a patient's early outcomes after the first chemotherapy cycle. Therefore, we can introduce early imaging examination of the primary lesion or systemic examination based on early warning of biomarker changes. It is of great benefit to discover distal metastases or new lesions.

Currently, cytokeratin-19 fragment 21-1 (CYFRA21-1) and carcinoembryonic antigen (CEA) are two widely researched biomarkers used together in monitoring the course of disease of NSCLC.

CEA, a glycoprotein that participates in regulating cellular progression, cellular recognition, and cell adhesion, is used as a biomarker of various malignant tumors globally [12]. An existing study proved that CYFRA21-1 is an early predictive indicator for chemotherapy efficacy of advanced NSCLC patients [13]. A retrospective study presented that the elevated serum CEA level may predict a dismal efficacy on NSCLC patients treated with the PD-L1 inhibitor [14]. Ardizzoni et al. [15] first assessed the effect of declined serum CYFRA21-1 and CEA levels on the prognosis of advanced NSCLC patients during chemotherapy. CEA and CYFRA21-1 (20% below baseline level; assessed after the second cycle of chemotherapy) work as reliable biomarkers for the efficacy evaluation. Likewise, a recent study illustrated that serum CYFRA21-1 and CEA expression levels serve as prognostic factors of advanced NSCLC [16]. Despite abundant relevant studies, the significance of change rates of CYFRA21-1 and CEA in predicting the efficacy of platinum chemotherapy has not been investigated yet. An earlier study found that the change rate of CYFRA21-1 before and after one cycle of chemotherapy can be used to evaluate the efficacy of chemotherapy, but the sensitivity and specificity need to be improved [13]. Hence, it is of dramatic significance to improve the sensitivity and specificity of early evaluation of tumors to chemotherapeutic drugs.

Hence, this study explored the effect of change rates of CYFRA21-1 and CEA before and after the first cycle of chemotherapy in predicting chemotherapy efficacy on IIIb/IIIc or IV stage NSCLC patients.

## 2. Materials and Methods

### 2.1. Collection of Patients' Information

Data of 103 advanced NSCLC patients who received chemotherapy from February 2018 to November 2020 in Zhejiang Provincial People's Hospital were retrospectively analyzed. All patients were diagnosed with stage IIIb/IIIc or IV NSCLC by histology or cytology. Eastern Cooperative Oncology Group performance status (ECOG PS) was 0-2. Patients received at least 2 cycles of first-line platinum doublet chemotherapy. The following patients were excluded in this study: patients who had EGFR mutation or ALK and ROS-1 rearrangement, patients who have brain metastasis signals or develop brain metastasis after imaging examination, patients with serious complications and/or uncontrolled basic diseases, and patients with complicated interstitial LC. This study had been approved by the Ethics Committee of Zhejiang Provincial People's Hospital and performed in accordance with the guidelines of the Helsinki Declaration.

### 2.2. Detection of CYFRA21-1 and CEA Levels and Calculation of Change Rates

Peripheral blood samples (5 ml) of NSCLC patients were collected a week before the first chemotherapy cycle and the second cycle, respectively. Corresponding serum was prepared. The levels of serum CYFRA21-1 and CEA were determined by radioimmunoassay (Cobas® 8000, Roche Diagnostic K.K., Tokyo, Japan, and Chemiluminescent Enzyme Immunoassay System LUMIPULSE® L2400, FUJIREBIO INC., Tokyo, Japan). Based on 95% confidence interval (CI) of Chinese common people, the critical value of normal serum CYFRA21-1 and CEA levels is 3.3 ng/ml and 3.4 ng/ml, respectively [17]. The change rate of serum CYFRA21-1 level was calculated by the following formula: (CYFRA21‐1 level after first chemotherapy–CYFRA21‐1 level before first chemotherapy)∗100%. The change rate of serum CEA level was calculated the same as CYFRA21-1.

### 2.3. Assessment of Chemotherapeutic Efficacy

After the second cycle of chemotherapy, the efficacy was evaluated according to the Response Evaluation Criteria in Solid Tumors (RECIST) version 1.1 [18]. Patients were evaluated with complete response (CR), partial response (PR), stable disease (SD), and progressive disease (PD). Patients evaluated with CR, PR, and SD were allocated into the disease control (DC) group, and others were in the PD group.

### 2.4. Statistical Analysis

Statistical analysis was conducted on SPSS 25.0 software. Categorical variables were presented as proportional numbers and percentages. Comparison between groups was subjected to the Chi-squared test or Fisher's accurate test. The Kolmogorov-Smirnov test was applied to evaluate the normality of continuous data distribution before statistical analysis. If data were subjected to near normal distribution, they were displayed as the mean ± standard deviation (SD). Comparison between groups was tested by an independent *t*-test. Otherwise, data were displayed as medians and interquartile range (*M* (P25, P75)) and comparison between groups was tested by the Mann-Whitney *U* test.

To determine the relationship between serum CYFRA21-1 and CEA levels and chemotherapeutic efficacy, all patients were classified into 2 groups by change rates of serum CYFRA21-1 and CEA levels. Patients' age, sex, ECOG PS score, weight loss, smoking, histological subtype, primary tumor location, clinical stages, and chemotherapeutic regimens were adjusted. A generalized linear model (GLM) and linear trend test were applied to determine whether the change rates of serum CYFRA21-1 and CEA are significantly correlated with chemotherapeutic efficacy. Moreover, a receiver operating characteristic (ROC) curve was drawn to assess the critical value of change rates of serum CYFRA21-1 and CEA in predicting efficacy. Sensitivity and specificity calculated by area under the curve (AUC) were applied to determine the performance of serum CYFRA21-1 and CEA on accurately recognizing patients with good therapeutic responses. To determine the optimal critical value of change rates of serum CYFRA21-1 and CEA of NSCLC patients with significant expected efficacy, we chose the point with the highest sensitivity and specificity in the ROC curve. The potential optimal cut-off rate of serum CYFRA21-1 and CEA levels was evaluated through screening patients with significant chemotherapeutic efficacy. All tests were two-tailed tests. *p* value less than 0.05 was referred to as statistically significant.

## 3. Results

### 3.1. Efficacy and Basic Characteristics of NSCLC Patients after Chemotherapy

After two cycles of chemotherapy, there were 92 patients in the DC group and 11 in the PD group. Patients received 2-6 cycles of chemotherapy, and most of them received gemcitabine plus cisplatin (GP) or gemcitabine plus carboplatin (GC) regimen. Basic characteristics of patients in two groups included age, sex, weight loss, ECOG PS score, smoking, histological type, primary tumor location, clinical stages, and chemotherapeutic regimens. The differences in basic characteristics were not statistically significant (*p* > 0.05) (see Table 1). As shown in Figure 1, change rates of serum CYFRA21-1 and CEA in the PD group were significantly higher than those in the DC group.

### 3.2. The Relationship between Change Rates of Serum CYFRA21-1 and CEA and Chemotherapeutic Efficacy

The relationship between change rates of serum CYFRA21-1 and CEA and chemotherapeutic efficacy is shown in Table 2. Patients were classified into 2 groups according to change rates of serum CYFRA21-A and CEA. In the subgroups with CYFRA21-1 and CEA change rates ≤ 0, cases of PD were 4 (5.6%) and 1 (1.8%), respectively. In the subgroups with CYFRA21-1 and CEA change rates > 0, cases of PD were 7 (22.6%) and 10 (21.7%), respectively. These patients responded poorly to chemotherapy. After confounding factors like age, sex, ECOG PS score, weight loss, smoking, histological type, primary tumor location, clinical stage, and chemotherapeutic regimens were adjusted, it was shown that change rates of serum CYFRA21-1 and CEA were inversely correlated with chemotherapeutic efficacy. Moreover, the lowest change rate of serum CEA was significantly correlated with favorable chemotherapeutic efficacy (*p* = 0.004; Table 2). The linear trend between change rates of serum CYFRA21-1 and CEA and chemotherapeutic efficacy is shown in Figure 2.

### 3.3. Evaluation of the Optimal Critical Value of Change Rates of Serum CYFRA21-1 and CEA and Their Efficacy in Predicting Chemotherapeutic Efficacy

To evaluate the optimal critical value of change rates of CYFRA21-1 and CEA in predicting chemotherapeutic efficacy, the ROC curve was used to analyze the highest point of specificity and sensitivity. As shown in Figure 3 and Table 3, AUC values (95% CI) based on the change rates of CYFRA21-1 and CEA were 0.71 (0.49-0.94) and 0.85 (0.69-1.00), respectively. After the confounding factors were adjusted, the optimal AUC (95% CI) in predicting early chemotherapeutic efficacy was 0.87 (0.71-1.00), *p* < 0.001.

## 4. Discussion

Early assessment of the sensitivity of tumors to drugs is of great significance to guide the following treatment. At present, there are intensive studies on serum biomarkers in predicting cancer treatment efficacy, while few studies look into corresponding markers that could predict the early efficacy of cancer treatment. This study revealed that change rates of CYFRA21-1 and CEA before and after the first chemotherapeutic cycle were negatively correlated with chemotherapeutic efficacy, and they held high diagnostic value in predicting the chemotherapy efficacy.

Chemotherapy has long been the major strategy for LC treatment, whereas a study displayed limited benefits of maintenance chemotherapy for elder patients with advanced NSCLC [19]. It was our focus to early predict patients' chemotherapeutic efficacy to adjust therapeutic regimens. A study manifested that early clearance of HE4 and CA125 can predict the platinum sensitivity and prognosis of ovarian cancer patients. Monitoring HE4 and CA125 during first-line treatment may help to predict platinum sensitivity and risk for progression and recurrence [20]. In our study, change rates of CYFRA21-1 and CEA were negatively correlated with chemotherapeutic efficacy after platinum chemotherapy. Moreover, several studies testified that elevated CYFRA21-1 and CEA levels are relevant to patients' dismal prognosis [21, 22]. However, few studies have been devoted to the change rates of these two serums. Another study showed that CEA and lactate dehydrogenase (LDH) levels can be applied to evaluate advanced NSCLC patients' response to platinum chemotherapy [23]. Change rates of serum CYFRA21-1 and CEA were independent predictive factors.

Studies of tumor biomarkers manifested that the sensitivity or specificity of a single marker is relatively low and cannot meet the clinical requirement. Determination of various markers meanwhile is recommended both theoretically and practically to increase the sensitivity and specificity.

A meta-analysis provided evidence to evaluate the clinical efficacy of CYFRA21-1 and CEA in NSCLC treatment [24]. In this study, the combination of CYFRA21-1 and CEA holds better diagnostic value compared to a single biomarker. In early squamous cell carcinoma (SCC), baseline CYFRA21-1 and CEA levels can distinguish patients who benefit from adjuvant chemotherapy [25]. Likewise, the change rates of CEA and CYFRA21-1 can effectively evaluate chemotherapeutic efficacy in the early stage. For patients with preassessed PD, review of primary lesions, metastases, and even full-body imaging examinations can be conducted after the first cycle. Once the imaging PD occurs, the treatment plan of the second line should be adjusted instantly, so as to avoid the patients continuing to use the ineffective chemotherapy plan in the second cycle and improve the antitumor effect.

On the whole, this study displayed that change rates of serum CYFRA21-1 and CEA levels could predict the efficacy of early chemotherapy on NSCLC patients. The clinical significance of this finding lies in the early prediction of the efficacy, the early detection of patients with progression, timely adjustment of subsequent treatment strategies, improvement of treatment efficacy, and reduction of unnecessary treatment costs and unnecessary adverse reactions. In the future, we will further explore the predictive effects of CYFRA21-A and CEA on patients' long-term clinical efficacy, second-line or multiline therapy, chemotherapy combined with targeted therapy, or immune checkpoint inhibitors in the early stage.

## Figures and Tables

**Figure 1:** Comparison of change rates of serum CYFRA21-1 and CEA of patients in two groups. (a) Change rate of serum CEA of patients in DC group (blue) and PD group (red). (b) Change rate of serum CYFRA21-1 of patients in two groups. ^∗^*p* < 0.05.

**Figure 2:** The relationship between change rates of serum CYFRA21-1 and CEA and disease progression. (a) The relationship between CEA change rate and RR (95% CL) for PD. (b) The relationship between CYFRA21-1 change rate and RR (95% CL) for PD.

**Figure 3:** ROC curve and AUC indicate the sensitivity and specificity of change rates of serum CYFRA21-1 and CEA predicting chemotherapeutic efficacy.

**Table 1:** Efficacy and basic characteristics of NSCLC patients after chemotherapy.

Variable	DC (*n* = 92)	PD (*n* = 11)	*p* value
Sex, *n* (%)			1.000
Female	25 (27.2)	3 (27.3)	
Male	67 (72.8)	8 (72.7)	
Weight loss, *n* (%)			0.417
Weight loss < 5%	80 (87.0)	8 (72.7)	
Weight loss ≥ 5%	12 (13.0)	3 (27.3)	
Cigarette smoking, *n* (%)			1.000
Nonsmoker	38 (41.3)	5 (45.5)	
Smoker	54 (58.7)	6 (54.5)	
Age, *n* (%)			1.000
Age < 65 years	67 (72.8)	8 (72.7)	
Age ≥ 65 years	25 (27.2)	3 (27.3)	
Primary tumor type by location, *n* (%)			0.522
Central type	39 (42.4)	3 (27.3)	
Peripheral type	53 (57.6)	8 (72.7)	
Histological type, *n* (%)			0.17
ADC	52 (56.5)	7 (63.6)	
SCC	35 (38.0)	2 (18.2)	
Large cell	5 (5.4)	2 (18.2)	
ECOG PS score, *n* (%)			0.144
PS ≤ 1	73 (79.3)	6 (54.5)	
PS = 2	19 (20.7)	5 (45.5)	
Chemotherapy regimen, *n* (%)			0.84
GP	49 (53.3)	6 (54.5)	
GC	14 (15.2)	3 (27.3)	
TC	7 (7.6)	0 (0.0)	
AD	8 (8.7)	1 (9.1)	
AC	13 (14.1)	1 (9.1)	
DP	1 (1.1)	0 (0.0)	
Clinical stage, *n* (%)			0.769
IIIb/IIIc	17 (18.5)	3 (27.3)	
IV	75 (81.5)	8 (72.7)	

Categorical data were described as proportional number (%), and the chi-squared test or Fisher's exact test was selected to compare the differences between the 2 groups. Abbreviations: DC = disease control; PD = progressive disease; ADC = adenocarcinoma; SCC = squamous cell carcinoma; ECOG = eastern conference oncology group; GP = gemcitabine and cisplatin; GC = gemcitabine and carboplatin; TC = paclitaxel and carboplatin; AD = pemetrexed disodium and cisplatin; AC = pemetrexed disodium and carboplatin; DP = docetaxel and cisplatin.

**Table 2:** The relationship between serum CYFRA21-1 and CEA and chemotherapeutic efficacy.

Variables	*n*	PD cases (%)	Crude		Model 1		Model 2	
			RR (95% CI)	*p*	RR (95% CI)	*p*	RR (95% CI)	*p*
CYFRA21-1 change rate								
≤0	72	4 (5.6)	1.0 (1.0, 1.0)	Ref.	1.0 (1.0, 1.0)	Ref.	1.0 (1.0, 1.0)	Ref.
>0	31	7 (22.6)	5.0 (1.3, 18.4)	0.017	4.9 (1.3, 19.2)	0.022	3.0 (0.7, 12.8)	0.129
Per IQR = 0.52			2.6 (1.3, 5.2)	0.005	3.1 (1.4, 6.8)	0.005	2.1 (0.9, 4.5)	0.068
CEA change rate								
≤0	57	1 (1.8)	1.0 (1.0, 1.0)	Ref.	1.0 (1.0, 1.0)	Ref.	1.0 (1.0, 1.0)	Ref.
>0	46	10 (21.7)	15.6 (1.9, 126.8)	0.010	16.5 (1.9, 142.3)	0.011	13.0 (1.4, 118.0)	0.023
Per IQR = 0.55			5.8 (2.3, 14.8)	<0.001	6.0 (2.2, 16.8)	0.001	5.5 (1.7, 17.5)	0.004

IQR: interquartile range; cases: the number of participants in processing; RR: relative risk; CI: confidence interval. Model 1: adjusted for age, ECOG PS score, gender, and primary tumor type by location. Model 2: model 1+CYFRA21-1 change rate+CEA change rate.

**Table 3:** The prediction of chemotherapeutic efficacy through change rates of serum CYFRA21-1 and CEA.

ROC model	AUC (95% CI)	SE	*p*
CYFRA21-1 change rate	0.71 (0.49-0.94)	0.11	0.001
CEA change rate	0.85 (0.69-1.00)	0.08	<0.001
Total	0.87 (0.71-1.00)	0.08	<0.001

Total indicates the combination of CYFRA21-1 change rate, CEA change rate, ECOG PS score, and age.

## Data Availability

Please contact the corresponding author with a reasonable request for the original experimental data and materials.
